# Computational Intelligence-Based Model for Exploring Individual Perception on SARS-CoV-2 Vaccine in Saudi Arabia

**DOI:** 10.1155/2022/6722427

**Published:** 2022-04-06

**Authors:** Irfan Ullah Khan, Nida Aslam, Sara Chrouf, Israa Atef, Ikram Merah, Latifah AlMulhim, Raghad AlShuaifan

**Affiliations:** Department of Computer Science, College of Computer Science and Information Technology, Imam Abdulrahman Bin Faisal University, Dammam 31441, Saudi Arabia

## Abstract

Countries around the world are facing so many challenges to slow down the spread of the current SARS-CoV-2 virus. Vaccination is an effective way to combat this virus and prevent its spreading among individuals. Currently, there are more than 50 SARS-CoV-2 vaccine candidates in trials; only a few of them are already in use. The primary objective of this study is to analyse the public awareness and opinion toward the vaccination process and to develop a model that predicts the awareness and acceptability of SARS-CoV-2 vaccines in Saudi Arabia by analysing a dataset of Arabic tweets related to vaccination. Therefore, several machine learning models such as Support Vector Machine (SVM), Naïve Bayes (NB), and Logistic Regression (LR), sideways with the N-gram and Term Frequency-Inverse Document Frequency (TF-IDF) techniques for feature extraction and Long Short-Term Memory (LSTM) model used with word embedding. LR with unigram feature extraction has achieved the best accuracy, recall, and *F*1 score with scores of 0.76, 0.69, and 0.72, respectively. However, the best precision value of 0.80 was achieved using SVM with unigram and NB with bigram TF-IDF. However, the Long Short-Term Memory (LSTM) model outperformed the other models with an accuracy of 0.95, a precision of 0.96, a recall of 0.95, and an *F*1 score of 0.95. This model will help in gaining a complete idea of how receptive people are to the vaccine. Thus, the government will be able to find new ways and run more campaigns to raise awareness of the importance of the vaccine.

## 1. Introduction

Coronavirus 19, also referred to as COVID-19 or SARS-Cov-2, is a new virus that was first officially reported on December 2019 in Wuhan, Hubei Province, China, in December 2019 and declared a pandemic by the World Health Organization (WHO) in March 2020. As of January 19, 2022, 335,515,088 confirmed cases of infected individuals were reported worldwide from 222 different countries and territories and 626,808 cases reported in Saudi Arabia [1]. This raised a global concern as the number of cases continued to mount and authorities imposed precautionary measures and lockdowns to curb the spread of this virus.

Many universities, laboratories, and pharmaceutical companies started their research on a possible cure for this virus. Companies from several countries have contributed to the launch of new vaccines to reduce the infection rate of SARS-CoV-2. By the end of 2020, many vaccines were awaiting the WHO approval to be distributed and commercialized. The variation in vaccines and the approaches used to create the formula raised concerns among the public about whether they should take the vaccine. The only major difference between the proposed vaccines was that some use mRNA, which guides the body cells to produce a harmless piece called the “spike protein” while others, like most vaccines, use a weakened or inactivated version of the virus [2]. An example of the variation in vaccines is that both Pfizer and Moderna (using mRNA) report that their vaccine's effectiveness shows 95% in preventing moderate-to-severe symptoms of COVID-19 [3], while AstraZeneca (using a weakened version of the virus) has an efficacy of 63.09% [4].

Individuals have diverse opinion and feelings such as fear and concern regarding the variation in vaccines available. Social media is one of the platforms where people expressed their feelings and views on this topic. This data could be utilized by policy makers and could help professionals to learn more about the people's perception in the Kingdom of Saudi Arabia (KSA) and predict their level of awareness and the approach that the Ministry of Health and the government should take to raise awareness. Therefore, we are attempting to develop a model to analyse individual perception related to the SARS-CoV-2 vaccine using Machine learning (ML), Deep Learning (DL), and Natural Language Processing (NLP).

The main contribution of this study is to collect and prepare an Arabic dataset for SARS-CoV-2 vaccination awareness tweets in KSA. In addition to developing an ML and DL model and applying it to predict the individual awareness of the vaccines in the KSA, it also helps decision makers decide what should be done to increase awareness. Furthermore, the motivation of the study was to explore the individual perception about the SARS-CoV-2 vaccination in KSA using the sentiment analysis.

The study is divided as follows.  Section 2 provides an overview of related studies.  Section 3 discusses the material and methods, data collection, preprocessing, exploratory data analysis, the proposed feature extraction techniques (TF-IDF and N-gram), machine learning classifiers (SVM, NB, and LR), and the optimization strategy. Furthermore, LSTM model with word embedding was also used to compare the performance of the ML and Deep Learning (DL) models.  Section 4 contains the experimental setup and the results.  Section 5 includes the discussion. Finally, Section 6 summarizes the conclusion, recommendation, and future work.

## 2. Related Studies

Social media Sentiment Analysis (SA) has been discussed widely in research area and considered as either binary-class or multiclass classification problem by many researchers as they aim to classify tweets into positive, negative, and neutral sentiments' classes [5]. Sentiment analysis of Twitter data has been carried out in various domains, such as for product review, identifying sarcasm, strategic management, and education [6–9]. Twitter is one of the most used platforms by social media users because it allows users to post and distribute tweets within a certain limit of characters and communicate with each other in real-time manner. Twitter plays a significant role in analysing people's opinions and emotions in any area and discovering relationships and trends in society. Analyzing Arabic data is considered to be one of the most challenging SA types because it contains a vast dictionary and complicated structure. In recent years, several studies have focused on the analysis of Arabic tweets.

During SARS-CoV-2, several studies related to the analysis of twitter data, including sentiment analysis, mental health identification, individual perceptions related to governmental policies, and fake news detection, were conducted [10]. Abdelminaam et al. [11] performed a comparative analysis of ML and DL techniques to identify the fake news about SARS-CoV-2 from English tweets. They found that the DL models, that is, Long Short-Term Memory (LSTM) and Gated Recurrent Unit (GRU), outperformed the ML models. In the section below, we examined the SA for tweets about different vaccination and then discussed the techniques for SARS-CoV-2 vaccination.

### 2.1. Sentiment Analysis on Tweets about Different Vaccination

The best way to fight any disease or virus is to stop it from spreading between people and help them build an immunity to the disease, and this is the greatest importance of vaccination as it helps humans to create antibodies' form to fight the disease in the future. Many studies have focused on analysing people's opinions and concerns about the vaccination processes.

Dredze et al. [12] have conducted a social media analysis in 2016 to study public opinion about the Zika virus vaccine. The dataset contains 150,000 tweets between January 1 and April 29, 2016, which were analysed using big data computational techniques and supervised ML models to identify the tweets that discussed pseudoscientific claims about the vaccination. The study showed that it is more challenging to change the society's opinion about any topic than to form a new one; 86% of users who discussed pseudoscientific claims about the Zika vaccine have discussed the vaccination earlier in 2015 and 19% of them delivered antivaccine messages.

Similarly, Yuan and Crooks [13] examined 660 thousand tweets gathered after the outbreak of Disneyland measles in 2015 in California to analyse Twitter users' opinion about measles, mumps, and rubella (MMR) vaccines and help the healthcare professionals bridge the gap of communication with people and to deliver them with the right information about vaccination. The study aimed to classify the collected tweets into 3 categories: antivaccination, neutral to vaccination, and provaccination using supervised learning techniques such as LR, NB, SVM (linear and nonlinear kernel), nearest centroid, and KNN along with TF-IDF feature extraction technique. Linear SVM has achieved the best results with an accuracy of 0.746. The study concluded that pro- and antivaccine users' only tweet and communicate with people who agree with them and belong to the same opinion group, but neutral opinions can be distributed between both groups; this also proved that it is difficult for health sector workers to penetrate Twitter users because they communicate through enclosed and clustered platform.

Zhou et al. [14] also analysed 42 thousand tweets between October 2013 and March 2014 in order to predict antivaccine tweets about human papillomavirus (HPV) vaccines using supervised ML techniques. In the study, 2150 tweets were manually labeled as antivaccine tweets or not by the researchers and used to train the classifiers after applying the N-gram feature extraction technique to them. SVM classifier was constructed using 10-fold cross-validation to create two models aimed at analysing the content of the tweets (content-based) and the relationships of the tweet's writer with other users on twitter (connection based). The classifier, which relied on social connection features, outperformed the other classifiers with an accuracy of 0.886, suggesting that people's connections on Twitter could give the health services sector more insight into Twitter users than what they wrote. Featherstone et al. [15] assessed the vaccination information on social media by analysing 14,735 influencers' tweets about childhood vaccines from July 1 to October 15, 2018, when it was the period of outbreak of the measles in Europe. The start of measles in the United States and beginning of school year was when parents need to provide their children's vaccination status for school entry. The study clustered the influencers into three communities: one antivaccine and two provaccines by using social network community detection. Analyzing the natural text was done by using semantic network analysis (SNA), and the chi-square test was used to assess the significance of the relative difference among the sentiment for each community and the result showed that the antivaccine community had the highest rate of negative sentiments and discussion more about the harms of vaccines, while the provaccine communities discussed vaccine prevention resulting in more positive sentiment.

Similarly, Mitra et al. [16] used 49,354 tweets collected over the four years 2012–2015 to explore the users' attitudes towards vaccination and applied N-gram feature extraction to them. The study used SVM and 10-fold cross-validation with a prediction accuracy of 84.7% to classify users into three cohorts: active-pro- and active-antiusers who persistently adopt pro- and anti-attitudes, and joining-antiusers who are newly adopt anti-attitude. Lexical approaches such as Meaning Extraction Method (MEM) and LWIC program to have been adopted to figure out people's opinions on the vaccination issue and what topics they mentioned. The study concluded that the veteran antivaccination group are persistent in their beliefs, distrust the government, and tend to conspiratorial worldviews and that the new anti-vaccination adoptees share the same conspiracy thinking. Thus, they tend to acquire their attitude and believe in vaccination myths. Therefore, alternatives to traditional approaches of using authoritative sources are needed, such as correcting misleading thoughts about vaccination claims.

Khandelwal and Salathe [17] conducted a study to analyse spatiotemporal sentiment towards influenza A (H1N1) vaccination by analysing 477,768 tweets between August 25, 2009, and January 19, 2010. The N-gram feature extraction technique was applied to the tweets and then classified into four groups: negative, positive, neutral, and irrelevant, using classifiers such as NB to classify the tweets into negative or positive tweets, and the Maximum Entropy (ME) classifier to discover the neutral and irrelevant tweets. The ME classifier was used when there was a conflict occurring in classifying the tweets and it achieved an accuracy of 0.842. A positive correlation was found between expected vaccination rates based on sentiments' tweets and vaccination rates estimated by the CDC.  Table 1 presents the sentiment analysis studies related to different virus vaccinations.

### 2.2. Sentiment Analysis on Tweets Related to SARS-CoV-2 Vaccination

Lyu et al. [18] studied the opinion of the general citizens on possible SARS-CoV-2 vaccines. A human-guided ML framework was used to collect the diverse public views on the vaccine from 40,000 rigorously selected tweets across the U.S. The tweets were then categorized into three different types: people who are willing to take the vaccine, others who have doubts, and others who are against it. In addition, a multinomial LR was used to compare between the three groups by inferencing different features such as demographics, income, political affiliation, and so on. The result of the study, with an overall accuracy of 0.63 and precision of 0.70, showed that people who had a terrible pandemic experience have higher antivaccine opinions, where people who struggle socioeconomically oppose opinions about the vaccine.

Furthermore, Alam et al. [19] proposed a Deep Learning model for the sentiment analysis of the SARS-CoV-2 vaccination using Kaggle tweet dataset. Initially the polarity of the tweets was calculated using the dictionary approach. They found that most of the tweets were neutral. For the classification, bidirectional LSTM was used and achieved an accuracy of 90.83. They found that North America has the highest number of people fully SARS-CoV-2 vaccinated. However, the highest number of tweets was from India.

Al-Mohaithef and Padhi [20] conducted a web-based survey to explore the SARS-CoV-2 vaccine acceptance in KSA. The survey was conducted across the four major cities in KSA. The sample size of 992 was used to analyse the acceptance. They found that 64.7% of the people were willing to take the SARS-CoV-2 vaccine. The LR model was used for the analysis. Furthermore, they found that age, marital status, and education are the significant features for the willingness of the SARS-CoV-2 vaccine. However, another study has used the combined approach, that is, the use of questionnaire and twitter data for exploring the SARS-CoV-2 vaccination hesitancy [21]. Conversely, they found that the number of negative tweets was higher, followed by the positive tweets and then the neutral tweets. The tweets were collected from July 1 to July 21. VADER was used for lexicon analysis while for ML-based sentiment analysis Microsoft Azure was used. They found that the number of positive tweets in the first week was higher while in the third week the number of negative tweets was higher compared to the positive and neutral ones. The short data collection period is one of the limitations of this study.

Additionally, Pristiyono et al. [22] used the NB algorithm for the sentiment analysis of the SARS-CoV-2 tweets in Indonesia. The tweets were collected from January 15, 2021, to January 25, 2021. Similarly, the study found that 56% of the tweets were negative. Like the previous study, it also suffers from the short data collection duration and keywords used to collect the data. Similarly, Nezhad and Deihimi [23] conducted the SARS-CoV-2 vaccination sentiment analysis in Iran. Persian tweets were collected for the duration of April 1, 2021, to September 30^,^, 2021, for different types of vaccines. The sentiment analysis was performed using the CNN-LSTM model. Furthermore, they performed the comparative analysis of the vaccine developed in home and the imported vaccine. They found that negative sentiments have increased with the passage of time. Also, the distribution of negative and positive tweets was the same overall.

Shamrat et al. [24] used KNN model for sentiment analysis of SARS-CoV-2 vaccine. The significance of the study is that they performed the sentiment analysis for different types of popular SARS-CoV-2 vaccines like Pfizer, Moderna, and AstraZeneca. Moreover, they found that Pfizer has the highest number of positive tweets (i.e., 47.29%); however, Moderna has 46.16% and then AstraZeneca has 40.08%. Recently, Fazel et al. [25] performed a study to explore the individual perceptions of SARS-CoV-2 in the UK using twitter data. The dataset was collected from November 2020 to January 2021. They found that the number of tweets in November 2020 was high because the SARS-CoV-2 vaccine trial was released during that time. However, with the passage of time, the number of tweets decreases. Similarly, after the approval of the SARS-CoV-2 vaccine, the number of tweets again increased. While during the Christmas season, it dropped significantly. The number of positive tweets was significantly higher than that of negative category. Hybrid technique was used that combine the ML and the rule-based approach to classification.

Conclusively, all previous studies have either focused on SA in general topics during SARS-CoV-2 pandemic or on vaccine-related analysis for earlier pandemics over the last century not specifically related to SARS-CoV-2 stand using ML approaches. As per the author's knowledge, there is no study so far conducted on sentiment analysis related to SARS-CoV-2 in KSA using Arabic tweets. Moreover, most researchers focused on analysing English tweets and neglected all other languages, leaving a large gap in the world's population unexplored or studied.

However, Table 2 presents the sentiment analysis studies related to vaccination against SARS-CoV-2 virus. It is obvious from Table 2 that studies related to SARS-CoV-2 vaccination are being conducted either before or after the availability of the vaccination. Nevertheless, in the current study, we included the tweets from before and after the vaccine became available. Furthermore, the previous study analysed English tweets. However, in the proposed study, we aim to conduct SA on Arabic tweets specifically in the Saudi Arabia region to discover Saudi's opinion about SARS-CoV-2 vaccine and raise the public awareness of the vaccination processes.

## 3. Material and Methods

To explore the individual perception related to SARS-CoV-2 vaccination, there is a need to collect the dataset. The data was collected from the social media platform Twitter. Prior to applying ML algorithms on the dataset, certain preprocessing steps were applied to clean the data. After preprocessing, the dataset was annotated, and later prediction model was developed using ML and DL.  Figure 1 illustrates the block diagram for the proposed study.

### 3.1. Dataset Collection

The dataset downloaded from the Twitter platform using Twint scraping tool [26]. The data was collected between August 10, 2020, and April 4, 2021. Only the tweets from the Kingdom of Saudi Arabia were considered. The keywords used to collect the tweets are as follows:

- “سم مو دوا” “لقاح كورونا” “لقاح الصيني” “حقل تجارب” “#فايزر” “فايزر” “تجارب لقاح” “تطعيم” “#لقاح” “تطعيمه” “#اللقاح_اولويه” “لقاح كورونا الجديد” “استازينيكا” “موديرنا” “تلقيح” “موامره كورونا” “تطعمت” “لقاح” “محنا مطعمين”
- لا للتطعيم” “لا للقاح” “ما بنتطعم” “ماباخذ اللقاح” “مابتلقح” “تطعيم يخوف” “لقاح يخوف” “تطعيم عقم” “وفاة تطعيم” “تطعيم جلطة” “لقاح جلطة”
- “التطعيم متاجره” “ارواح الناس تطعيم” “خايف اطعم” “خايف اتطعم” “لا+_للتطعيم” “رافض للتطعيم” “ارفض التطعيم”“معارض للتطعيم” “ما ابي اطعم”
- “اخاف لقاح” “تطبيل لقاح” “اثار لقاح” “مضاعفات لقاح” “لقاح سام” “لقاح خطير” “لقاح خطير” “اموت لقاح” “تناقض لقاح” “ترويج لقاح” “رافض لقاح” “معارض للتطعيم” “عدم اللقاح”
- “اخاف لقاح” “تطبيل لقاح” “اثار لقاح” “مضاعفات لقاح” “لقاح سام” “لقاح خطير” “لقاح خطير” “اموت لقاح” “تناقض لقاح” “ترويج لقاح” “رافض لقاح” “معارض للتطعيم” “عدم اللقاح”
- “لقاح اجبراي” “تناقض لقاح” “لقاح تجلط” “تعطيم مضر” “تعطيم تجلط” “لقاح مضر” “لقاح جلطة” “تعطيم زعل” “لقاح موت” “تطعيم موت” “تطعيم جلطة” “لقاح عقم” “تطعيم عقم” “ترويج لقاح” “رافض تطعيم” “عدم اللقاح”
- “Poison Not a cure” “Covid Vaccine” “Chinese Vaccine” “Experimental Field” “Pfizer” “Vaccine Experiments” “Vaccination” “#Vaccine” “Vaccine Priority” “New Covid Vaccine” “Astrazeneca” “Moderna” “vaccination process” “Covid's conspiracy” “I am vaccinated” “vaccine (different synanon)” “We are vaccinated”
- No to vaccination” “No to the vaccine” “We do not receive the vaccine” “Do not get vaccinated” “Don't be vaccinated” “Vaccination fear” “Vaccines fears” “sterility” “death of vaccination” “vaccination clot”
- “Vaccination is a trade.” “People's lives, vaccine” “I am afraid to be vaccinated” “I am afraid to be immunized” “No +_ to vaccination” “Refuse to be vaccinated” “I refuse to be vaccinated” “I am against vaccination” “I do not want to be vaccinated”
- “I am afraid of a vaccine” “overestimating vaccine” “vaccine effects” “vaccine complications” “toxic vaccine” “dangerous vaccine” “dangerous vaccine” “I will die of a vaccine” “vaccine contradiction” “vaccine promotion” “vaccine refusal” “opposition to vaccination” “not vaccinated”
- forced vaccine” “contradictory vaccine” “clotting vaccine” “harmful vaccination” “clot vaccination” “harmful vaccine” “clot vaccine” “disturbing vaccination” “death vaccine” “death vaccination” “clot vaccination” “sterility vaccine” Sterility vaccination “vaccine promotion” “vaccination refusal” “no vaccination”

Initially, the number of tweets collected was 10991. Some of the tweets were initially removed since they were duplicate, irrelevant, contain only link, and so on. After initial preprocessing, 3000 tweets were used for annotation. Since the aim of the study is to explore individual perceptions related to SARS-CoV-2, all tweets were manually annotated into 3 distinct classes: provaccination, neutral, and antivaccination. In the dataset, neutral tweets exceeded both provaccination and antivaccination with 1492 tweets. After that, provaccination class with 1153 tweets, and finally antivaccination class with the lowest number of tweets of 355.  Figure 2 shows the number of tweets per class label.

### 3.2. Preprocessing

One of the most critical challenges in analysing the Arabic text is the data preprocessing and cleaning due to the complex structure of the Arabic language and the variety of the homonym vocabulary in its dictionary. Moreover, Twitter tweets usually contain noisy data, such as links, pictures, videos, nontextual symbols, and emojis. Consequently, the data corpus requires intensive cleaning and preprocessing before being fed into an analysis model to get the best and desired results.

During the preprocessing phase, the following techniques were applied:

- Remove links and pictures
- Remove nontextual data, such as hashtags, mentions, punctuations, and emojis
- Remove stop-words: stop-words are the phrases that do not affect the meaning of the sentence and have no huge value in it and have no impact such as “و,” “إلى,” “عن,” and “على”
- Remove Arabic vocalization (Tashkeel): Arabic language has special symbols that may affect the words interpretation by ML models (“َ,” “ ٍ,” “ٌ”)
- Remove repeated characters in the same words: (“قااال”) will be (“قال”)
- Tokenization: break each sentence to integral parts called tokens

### 3.3. Feature Selection

The performance of the ML algorithms depends upon features used to train the model. Similarly, the classifiers perform better with the numbers than with the text. Therefore, there is a need to apply feature extraction and selection techniques to transform the textual data into numeric vectors that could be better manipulated by the classifiers. In this study, we aim to apply two widely used techniques for selecting textual data features. Firstly, N-gram technique is considered, which helps in finding the relationship between adjacent words in a text and the possibility that they occur together. N represents the number of adjacent words considered as a sequence. In the unigram, each word is considered as a single sequence, whereas in bigram every two words are a sequence [27, 28].

Secondly, the Term Frequency-Inverse Document Frequency (TF-IDF) technique is applied in combination with unigrams and bigrams to study their impact on models' performance. The TF-IDF technique focuses on giving high weights to the words that contribute more to the text meaning and neglect or assign low weightage to nondiscriminative words and phrases.

The TF-IDF is a method to evaluate the importance of a word (token) in the document. Term frequency calculates how many times the word exists in the document, and inverse document frequency calculates the number of documents in which the word exists. TF-IDF is a method to transform the textual representation of data into a Vector Space Model (VSM). Representing documents as vectors is the fundamental for retrieving information from scoring documents in a query. A query (*q*) is viewed as a bag of words and can be treated as a very short document, which can also be viewed as a vector. The assigned score to each document is equal to the dot product of the document and the query.

(1) $$\begin{array}{c} \overset{⟶}{v}\left(q\right)\cdot \overset{⟶}{v}\left(d\right). \end{array}$$

The score of the document for a specific query is considered as similarity between the query vector and the document vector.

(2) $$\begin{array}{c} \text{score}\left(q,d\right)=\;\frac{\overset{⟶}{v}\left(q\right).\overset{⟶}{v}\left(d\right)}{\left|\overset{⟶}{v}\left(q\right)\right|\left|\overset{⟶}{v}\left(d\right)\right|}. \end{array}$$

### 3.4. Exploratory Data Analysis

Exploratory analysis of the dataset was performed to gain initial insight into the downloaded tweets. The tweets were manually labeled.  Table 3 contains some of the samples of the manually annotated tweets.

Figure 3 shows the length of the tweets for the complete dataset (pro-, anti-, and neutral vaccination). Most tweets were 35–70 words long. Furthermore, Figures 4 and 5 represent the top 10 and 20 unigrams and bigrams in the dataset.

## 4. Description of the Classifiers

### 4.1. Logistic Regression

Logistic Regression (LR) is one of the widely used supervised ML algorithms for classification of binary and multiclass problems [29]. LR showed significant outcomes at classifying simple data sets that are linearly separable, but it may require regularization techniques for high-dimensional data. LR models use the mathematical logistic function, which can be described as follows:

(3) $$\begin{array}{c} F\left(z\right)=\frac{1}{\left(1+e^{-z}\right)}. \end{array}$$

The function output ranges between 0 and 1. The output of the function describes the probability of getting a certain class target for the dependent variable.

Logistic regression is widely used in analysing binary outcomes. It is like linear regression, but it is more complicated to evaluate it graphically. The training process depends on choosing the parameters; the parameters should define the function that maximizes the posteriori likelihood function [30]. For example, let C be the number of classes identified as *C*  ∈  {1,2,…, *C*}, and let *X* be the feature vector of length *n*. Thus, the given equation (4) represents the probability that *X* belongs to one of the *C* classes. *C*  ∈  {1,2,…, *C*} represents the parameter vectors that define regression coefficients, and 〈.,.〉is the vectors inner product.

(4) $$\begin{array}{c} \mathrm{Pr}\left(Y=k|x\right)=\frac{e^{\langle \beta_{k},X\rangle }}{\sum_{i=1}^{K}e^{\langle \beta_{i},X\rangle }}\text{ for }k=1,2,\ldots ,k. \end{array}$$

From the training process, the coefficient *β*_*k*_ can be obtained. Then, equations (5) and (6) will be used to predict the outcome of feature vector *X* [12].

(5) $$\begin{array}{c} k^{*}\in \arg\max\mathrm{Pr}\left(Y=k\left|X\right|\right),\;k\in \left\{1,2,\ldots ,K\right\}, \end{array}$$

(6) $$\begin{array}{c} k^{*}\in \arg\max\langle \beta_{x},X\rangle ,\;k\in \left\{1,2,\ldots ,K\right\}. \end{array}$$

### 4.2. Support Vector Machine

Support Vector Machine (SVM) is a supervised ML algorithm used for regression, classification, and features selection [31]. SVM models work on the principle of finding the optimum hyperplane that separates the data classes from any other high-dimensional feature space.

SVM separates the classes by a linear function. The linear function of SVM is as follows.

(7) $$\begin{array}{c} f\left(x\right)=\mathrm{sgn}\left(w\cdot x+b\right). \end{array}$$

As *w* is weight for the support vectors, *x* represents the features that are inputted to SVM, and *b* is the bias. Also, selecting the optimal separating hyperplane in SVM depends on the maximum margin for the concept of hyperplane, where the margin represents the distance between the nearest support vector and the hyperplane that maximizes the ability of SVM prediction to classify new examples correctly.

SVM works by using a decomposition toward scalar products and support vectors which are presented in a kernel form. SVM works on linear data and nonlinear data. In linear problems, simple hyperplane can be used to separate the data while for nonlinear data a kernel function should be addressed to map the data into higher-dimensional feature space. However, the training time is huge for SVM classifier due to huge number of parameters in the model.

### 4.3. Naive Bayes

Naive Bayes (NB) is a probabilistic classifier that assumes no relationship or dependency between all the input features and relies on a linear model [29]. Although real-life problems usually contain dependency between input features, NB shows significant results compared to other classifiers specifically in text classification. NB computes the probability of the target class given an input feature based on Bayes' rule. Unlike the standard Naïve Bayes that is the conditional independence of each feature in the model, the Multinomial Naïve Bayes model considers the multinomial distribution for each feature in the model. When calculating the probability of observing *f*_1_ through *f*_*n*_ features, given some class *c*, the Naïve Bayes assumption holds:

(8) $$\begin{array}{c} p\left(f_{1},\;\ldots ,\;f_{n}|c\right)=\;\prod_{i=1}^{n}p\left(f_{i}|c\right). \end{array}$$

The probability of classifying a new example with the Naïve Bayes model will work simply as follows:

(9) $$\begin{array}{c} p\left(c|f_{1},\;\ldots ,\;f_{n}\right)\propto p\left(c\right)p\left(f_{1}|c\right)\ldots p\left(f_{n}|c\right). \end{array}$$

The difference is that Multinomial Naïve Bayes gives information about each *p*(*f*_*i*_*|c*) as a multinomial distribution, rather than some other distributions.

### 4.4. Deep Learning Model

In addition to machine learning algorithms, we have used the word embeddings to train a deep neural network based on a Long Short-Term Memory (LSTM) unit [32]. LSTM is a sophisticated version of RNN used for sequential modelling and it does not suffer from the vanishing gradient problem. LSTM is designed to circumvent the dilemma of long-term dependency. Retaining knowledge over time is particularly their default response. LSTM is intended to estimate the conditional probability *p*(*y*_1_,…*yT* ′*|x*_1_,…*xT*), where (*x*_1_,…*xT*) is an input sequence and (*y*_1_,…*yT* ′) is corresponding output sequence. The LSTM computes this conditional probability by first obtaining the fixed dimensional representation vector of the input sequence, and then computing the probability using a standard LSTM-LM formulation. For this purpose, an embedding model based on FastText Word2Vec model, that is, arabic-news.bin, with a vocabulary size set of 2000, a maximum input sequence length set of 60 tokens, and a vector size of 300 in the final embedding matrix is used. The structure of the model was based on the sequential Keras API, where the first layer is an embedding layer with parameter settings like max_vocab_size = 2000, embed_dim = 256, and input_length = 60. The 2nd layer comprises an LSTM layer with 196 cells that have Dropout = 0.2 and Recurrent_dropout = 0.2. Two dense layers were added with 128 and 64 neurons with “ReLu” as the activation function, while the last layer contains 3 neurons based on the number of classes with “softmax” activation function. The model configuration setting includes optimizer = “Adam,” loss = “categorical_crossentropy,” and matrics = “accuracy.” To train the model, the number of epochs was set to 10 with batch_size = 64.

### 4.5. Optimization Strategy for ML Models

SVM and LR classifiers have different parameters that affect the performance of the models such as Gamma, and kernel for SVM and Solver, *C*, and penalty for LR. However, Naïve Bayes model does not contain any parameters, so no optimization was performed. In order to get the best parameters for these models, Grid Search parameter tuning technique is used. Grid Search works in brute force manner and tests all the combinations of the possible parameters to get the best parameters collection for the model. Tables 4 and 5 represent the optimum parameters for SVM and LR.

## 5. Experimental Setup and Discussion

The models were implemented using Python version 3.9.2. In this study, we used three ML classifiers along with multiple variations of N-grams and TF-IDF features extraction techniques to predict peoples' sentiment and opinion related to SARS-CoV-2 vaccination. In addition, LSTM model with embedding feature extraction was also used. The evaluation measures used in our study were accuracy, precision, recall, and *F*1 score. Since our dataset contains imbalanced classes, therefore we focused more on precision, recall, and *F*1 score. These measures provide better insight into the nature of the predicted outcome.

Initially the experiment was conducted using unigram and bigram without IF-TDF for all the implemented classifiers. Later, the experiment was conducted using uni- and bigram with IF-TDF. Due to the imbalanced classes in the dataset, stratified splitting was applied to ensure that the training and testing sets get sufficient records of each class. The training set contains 80% (2400 tweets) of the dataset whereas the remaining 20% (600 tweets) were used for testing.  Table 6 summarizes the results of the experiments using proposed models.

From the experimental results above, it can be seen that LR with unigram gave the best accuracy, recall, and *F*1 score results with values of 0.76, 0.69, and 0.72, respectively. SVM with unigram TF-IDF showed very competitive and close results to LR and it gave the best precision value of 0.80. On the other hand, NB with bigram TF-IDF showed the worst accuracy, recall, and *F*1 score but it presented good precision value. Overall, it is concluded that unigram feature extraction, either with TF-IDF or without, gave best performance with all the classifiers. Moreover, LR and SVM showed good results compared to NB, which in some cases had a very weak prediction. Figures 6 and 7 show the confusion matrices for the best-performing models: LR with unigram and SVM with unigram TF-IDF, respectively. However, the LSTM model outperformed the results achieved by the ML models in terms of all evaluation measures. The model achieved similar accuracy, recall, and *F*1 score of 0.95, while the precision was 0.96. The results have shown the significance of LSTM in the prediction of individual perception on SARS-CoV-2 vaccine.  Figure 8 shows the confusion matrix for the LSTM model. Furthermore, Figure 9 contains the ROC (Receiver Operating Characteristic) curve for the LSTM model.

## 6. Discussion

During the study, we initially found a total of 10991 retrieved tweets and after the preprocessing 3000 relevant tweets were selected and annotated. The tweets were collected between August 10, 2020, and April 4, 2021, the duration of the tweets collection was 9 months. From the collected tweets, it has seen that people in KSA are usually either provaccination (positive class) or neutral, while very few people are against vaccination that is around 12% of the tweets in the dataset. Furthermore, the number of neutral tweets in the current dataset is 49.7% similar to that of Alam et al. [19] and also contains the least number of tweets related to the negative perception of the SARS-CoV-2 vaccines. Similarly, Al-Mohaithef and Padhi [20] explore the acceptance of the SARS-CoV-2 vaccine in KSA using the questionnaire approach and found that 64.7% of people accept the vaccination from four main cities of KSA. However, the number of positive tweets in the proposed study is less than [20] as the data collected in the current study was from Twitter but Al-Mohaithef and Padhi's [20] study only focused on the data from the main cities of KSA. Furthermore, samples were collected from individuals with at least postgraduate qualification.

Conversely, Roe et al. [21] analysed the data collected via questionnaires and tweets and found a higher number of negative tweets when compared with the positive ones. However, the data collection was made in July 2021 and during that time vaccine has already been introduced and most of the countries have already imposed the SARS-CoV-2 vaccination. The main limitation of the study was the short duration of data collection. Likewise, Pristiyono et al. [22] also suffered from the short data collection duration, which is one week from January 15, 2021, to January 22, 2021. During this period, SARS-CoV-2 vaccination was simply introduced; hence, the number of negative tweets was very high when compared to positive and neutral classes. The tweets were collected from Indonesia. Moreover, the tweets from the UK were analysed in Fazel et al.'s [25] study and they found that the number of negative tweets was high when the vaccination trials were introduced, but with the passage of time, the intensity of the tweets was reduced. Most of the tweets analysed in the previous study have a short data collection duration. While in the current study, the data was collected for a period of about 9 months. However, our study also suffers from some limitations. They have broadly collected and analysed the data from the KSA. There is a need to specifically analyse the data from different regions of KSA and explore the sentiment trends at the time of major announcement from the Government of KSA related to SARS-CoV-2 vaccination. Furthermore, the size of the dataset is limited.

## 7. Conclusion and Recommendation

This study aims to measure the Saudis' acceptance of SARS-CoV-2 vaccines and their knowledge and the importance in limiting and controlling the spread of the virus. The study implemented three ML classifiers: SVM, LR, and NB and DL models; that is, LSTM aims to predict the awareness of Twitter users toward the vaccination process in Saudi Arabia. LSTM outperformed the ML models with an accuracy, recall, and *F*1 score of 0.95 and a precision of 0.96. While in ML models, LR with unigram feature achieved the best accuracy with a value of 0.76, recall with a value of 0.69, and *F*1 score with a value of 0.72, whereas SVM achieved the best precision with value of 0.80. The results of this study can help authorities and decision makers to set a suitable plan to encourage more people to get vaccinated. For future work, we recommend extending the work by adding aspect-based mining on SARS-CoV-2 vaccines, also using other social media platforms to measure awareness. Furthermore, there is a need for a multilingual sentiment analysis tool for covering languages like Urdu, French, Italian, and others. This will help in increasing the global awareness about the vaccines around the world, thus reducing the global spread of the virus.

## Figures and Tables

**Figure 1:** Block diagram for the proposed methodology.

**Figure 2:** Distribution of tweets per class in the dataset.

**Figure 3:** Distribution of number of sample and the length of the tweets in the dataset.

**Figure 4:** Distribution of top 10 unigrams after preprocessing.

**Figure 5:** Distribution of top 10 bigrams after preprocessing.

**Figure 6:** Confusion matrix for logistic regression.

**Figure 7:** Confusion matrix for support vector machine.

**Figure 8:** Confusion matrix for LSTM model.

**Figure 9:** LSTM model ROC curve for the three classes.

**Table 1:** Summary of previous studies related to different vaccination.

Ref	Dataset	Number of tweets	Language	Virus	Feature extraction	Technique	Accuracy
[12]	Tweets collected from Twitter	150,000	English	Zika	—	Descriptive analysis	—
[13]	Tweets collected from Twitter	660,000	English	Disneyland measles	TF-IDF	SVM	0.746
[14]	Manually collected	2150	English	HPV	N-gram	SVM	0.886
[15]	Tweets collected from Twitter	14735	English	Measles	—	SNA, chi-square	—
[16]	Tweets collected from Twitter	49,354	English	Newborn vaccinations	N-gram	SVM	0.847
[17]	Tweets collected from Twitter	477,768	English	Influenza A (H1N1)	N-gram	ME	0.842

**Table 2:** Summary of previous studies related to SARS-CoV-2 vaccination and supervised sentiment analysis.

Ref	Dataset	No. of tweets	Language	Feature extraction	Technique	Accuracy
[18]	Tweets collected from Twitter	40,000	English	—	LR	0.63
[19]	Kaggle (tweets)	125,906	English	Word embedding	Bi-LSTM	0.98
[22]	Tweets collected from Twitter	6,000	English	—	NB	—
[23]	Tweets collected from Twitter	803,278	Persian	—	CNN-LSTM	—
[24]	Tweets collected from Twitter	10,000	English	—	KNN	—

**Table 3:** Sample tweets from each class.

Sentiment	Tweets sample in Arabic	Tweets translation to English
Provaccination	يوم امس اخذت الوالده الجرعه الاولي لقاح كورونا اسال الله ينفع ويحفظها الاهم روعه التنظيم والتنسيق والترتيب والسرعه والحفاوه والاهتمام والاحترافيه للجميع سعوديين ومقيمين شيء مشرف يستحق المديح والتقدير الحمدلله نعمه السعوديه وبلا مجامله	Yesterday, my mother took the first dose of the vaccine, May Allah protect her. Everything was well arranged, clean and professional. I thank God to be living in Saudi Arabia
	اسال الله العظيم ان يجعلها لقاح العافيه ويحميك شر وجميع الشعب	
Antivaccination	ما عمري تطعمت لان عندي فوبيا الابر وايد يقولون تطعموا وحاشتهم انفلونزا قويه يعني ما استفادو	I have not been vaccinated because I have a phobia of needles. Everyone who got vaccinated has a strong flu, so they did not benefit of it. After the introduction of the corona vaccine, mysterious deaths raise doubts
	طرح لقاح كورونا وفيات غامضه تثير الشكوك	
Neutral	يوم عظيم للبشريه فايزر تعلن لقاحها وارتفاع مؤشرات الاسواق والمال والاعمال واسعار النفط وشركات الطيران العالم يتعافي	Good day, Pfizer has announced their vaccines and obvious indication of rise in the market price and oil price and airlines, your excellency the minister of health all countries are signing contracts to get the vaccines. Will Saudi Arabia get it soon?
	معالي الوزير افاده للشعب اذا الحكومه وقعت اتفاقيات شراء لقاحات شركه فايز شركه موديرنا الامريكيه اغلب الدول تتسابق لشراء اللقاحات بعقود مسبقه افيدونا جزاكم الله خير	

**Table 4:** Optimum parameters for the proposed SVM model.

Parameters	Optimal value chosen
*C*	1
Gamma	0.1
Kernel	Linear

**Table 5:** Optimum parameters for the proposed LR model.

Parameters	Optimal value chosen
*C*	100
Solver	Liblinear
Penalty	*l*2

**Table 6:** Performance measure of classifiers using different features' extraction.

Model	Feature extraction and selection	Accuracy	Precision	Recall	*F*1-score
SVM	Bigram with TF-IDF	0.73	0.79	0.62	0.66
	Bigram without TF-IDF	0.74	0.74	0.67	0.7
	Unigram with TF-IDF	0.75	**0.80**	0.68	0.71
	Unigram without TF-IDF	0.73	0.74	0.67	0.7
NB	Bigram with TF-IDF	0.66	**0.8**	0.5	0.49
	Bigram without TF-IDF	0.72	0.66	0.68	0.67
	Unigram with TF-IDF	0.67	0.79	0.51	0.5
	Unigram without TF-IDF	0.69	0.69	0.67	0.68
LR	Bigram with TF-IDF	0.73	0.78	0.67	0.71
	Bigram without TF-IDF	0.72	0.73	0.64	0.67
	Unigram with TF-IDF	0.72	0.75	0.62	0.65
	Unigram without TF-IDF	**0.76**	0.72	**0.69**	**0.72**
LSTM model	Embedding techniques	**0.95**	**0.96**	**0.95**	**0.95**

## Data Availability

The dataset will be available from the corresponding author upon request.
